The article "A Case Found to Be Severe Acute Respiratory Syndrome Coronavirus 2 Positive Immediately Before Hospitalization for Infectious Mononucleosis" was published in 2021. Journal: Cureus.

# A Case Found to Be Severe Acute Respiratory Syndrome Coronavirus 2 Positive Immediately Before Hospitalization for Infectious Mononucleosis

**DOI:** 10.7759/cureus.19344

**Published:** 2021-11-08

**Authors:** Ryo Kawaura, Ryo Utakata, Daikei Kondo, Takanori Wakaoka, Masami Ohnishi

**Affiliations:** 1 Department of Head and Neck Surgery-Otolaryngology, Ogaki Municipal Hospital, Ogaki, JPN

**Keywords:** coinfection, epstein-barr virus, sars-cov-2, covid-19, infectious mononucleosis

## Abstract

The cases of coronavirus disease 2019 (COVID-19) mainly present with symptoms such as persistent fever, cough, and general malaise, which may become severe or fatal; while young people do not show these typical symptoms and are asymptomatic, some cases are infected with minor symptoms or none. Herein, we report a case of a 20-year-old woman who was hospitalized for infectious mononucleosis (IM). Initially, fever and sore throat were observed without typical COVID-19 symptoms, but polymerase chain reaction (PCR) tests performed before admission confirmed severe acute respiratory syndrome coronavirus 2 (SARS-CoV-2) positivity. Fortunately, she was discharged without any serious symptoms as IM and COVID-19. Virological examination suggested a primary infection with the Epstein-Barr virus. In the COVID-19 pandemic, we should also pay attention to the possibility of SARS-CoV-2 coinfection in mild and asymptomatic young cases, even if the symptoms suggesting IM are preceded.

## Introduction

The novel severe acute respiratory syndrome coronavirus 2 (SARS-CoV-2) is still prevalent worldwide, even in the latter half of 2021. Currently, with the spread of the 2019 coronavirus disease (COVID-19) vaccinations for the elderly and patients with preexisting illnesses, cases among young individuals who are undervaccinated are relatively increasing but do not exhibit typical COVID-19 symptoms such as high fever, cough, and general malaise. Herein, we report a case of a young woman who was hospitalized for infectious mononucleosis (IM). Despite the patient presenting only a few of the typical COVID-19 symptoms, polymerase chain reaction (PCR) performed before admission showed SARS-CoV-2 positivity. Although there are some reports of Epstein-Barr virus (EBV) reactivation due to SARS-CoV-2 infection [1-4], there are few reports on the co-occurrence of COVID-19 and IM [5,6].

## Case presentation

A 20-year-old woman with no medical history visited our hospital with complaints of sore throat and decreased oral intake. She is a student living with her parents and had been working part-time at a restaurant. She had been aware of the sore throat eight days before she visited our department. She consulted a nearby doctor three days after the onset of the symptoms who diagnosed her with tonsillitis and prescribed amoxicillin. The treatment was continued at home, and she stopped going to work and school. Nevertheless, the sore throat symptoms did not improve; hence, her former doctor added ceftriaxone infusion to her treatment. However, the sore throat and poor oral intake persisted; hence, she was referred to our department.

At the first visit, the patient did not exhibit trismus. She had mildly swollen bilateral palatine tonsils and redness of the soft palate. She had no asymmetrical tonsillar swelling but had mild impetigo on her tonsils; nevertheless, pseudomembrane-like white moss formation was not noted. The cervical lymph nodes were mildly enlarged. Her temperature was 37.2°C at the first examination. At the time, biochemical tests showed considerably increased serum aspartate aminotransferase (AST) and alanine aminotransferase (ALT) levels (141 vs. 148 U/L). By contrast, the serum C-reactive protein (CRP) level was 0.15 mg/dL, which was not significantly raised. The white blood cell count was 8420/µL, with neutrophil accounting for 29.0% and lymphocyte for 53.0%. Furthermore, the patient had an atypical lymphocyte proportion of 10.0%, which was an elevated value (Table 1). The patient also underwent laryngeal endoscopy (Figure 1a, 1b), during which we used standard personal protective equipment such as surgical masks, gloves, and face shields. The results showed swelling of the posterior third of the tongue but no laryngeal edema. Chest radiography also showed no apparent abnormal findings, such as infiltration shadows and consolidative changes (Figure 2).

**Table 1:** Results of the blood test at the initial visit The values given inside brackets mean the normal value in our department. T-Bil: total bilirubin, AST: aspartate aminotransferase, ALT: alanine aminotransferase, LDH: lactate dehydrogenase, γ-GTP: gamma-glutamyltransferase, ALP: alkaline phosphatase, TP: total protein, BUN: blood urea nitrogen, CRP: C-reactive protein, WBCs: white blood cells, RBCs: red blood cells.

Biochemistry				Peripheral blood			
T-Bil	0.3	mg/dL	(0.2-1.2)	WBCs	8,420	/μL	(3,500-9,900)
AST	141	U/L	(5-40)	Neutrophil	29	%	(38.0-75.0)
ALT	148	U/L	(3-35)	Lymphocyte	53	%	(16.5-49.5)
LDH	333	U/L	(124-222)	Monocyte	6	%	(2.0-10.0)
γ-GTP	33	U/L	(<56)	Eosinophil	1	%	(0.0-8.5)
ALP	66	IU/L	(38-113)	Basophil	1	%	(0.0-2.5)
TP	7.5	g/dL	(6.5-8.2)	Atypical lymphocyte	10	%	(0)
Albumin	4.1	g/dL	(3.5-5.0)	RBCs	414	×10^4^/μL	(353-484)
BUN	8.6	mg/dL	(8.0-23.0)	Hemoglobin	12.3	g/dL	(11.0-14.8)
Creatinine	0.71	mg/dL	(0.40-0.78)	Hematocrit	37.6	%	(31.4-43.1)
Glucose	149	mg/dL	(70-110)	Platelets	20.4	×10^4^/μL	(12-40)
CRP	0.15	mg/dL	(<0.25)				

**Figure 1:** Images of endoscopy Bilateral grade II tonsils of the Mackenzie classification with erythema of the soft palate were observed (a). There was no asymmetrical tonsillar swelling, and a small amount of pus was observed on the tonsils, but no white moss formation as much as pseudomembrane was observed (yellow allows). Laryngeal endoscopy showed swelling of the tonsils (yellow allows), but no laryngeal edema (b).

**Figure 2:** Chest X-ray Chest X-ray showed no abnormal findings such as obvious infiltration shadows or consolidative change. R: right side.

Based on the pharyngeal findings and blood examination results, we suspected IM. The patient was hospitalized due to her decreased oral intake. We conducted additional tests for related viruses such as EBV. She had no COVID-19 symptoms other than fever and sore throat; nevertheless, the patient had fever prior to hospitalization because the re-emergence of COVID-19 had not yet converged locally. She was moved from the outpatient department because of fever, and PCR was performed on a nasopharyngeal swab sample. The results showed that the patient was SARS-CoV-2 positive. Based on these results along with IM, she was admitted to the hospital for follow-up with only intravenous fluids in the isolation ward. In addition, because the patient needed to be isolated, the extent of hepatosplenomegaly could not be assessed on abdominal ultrasonography.

On day three of hospitalization, the sore throat improved and oral intake was good with no abdominal symptoms suggesting worsening of hepatosplenomegaly; hence, the infusion was terminated. On day four, a blood sampling test showed that the serum AST and ALT levels were 90 and 131 U/L, respectively, indicating that the elevated liver enzyme levels also improved. On day five, she developed an itchy rash all over her body, which disappeared by day seven following treatment with an antihistamine (fexofenadine). She did not exhibit toe redness, which is occasionally noted among COVID cases. Throughout her hospitalization, she did not have fever exceeding 38°C, and she was able to maintain oxygen saturation above 90% without the need for oxygen administration. On day 11, the patient was discharged 10 days after her first positive PCR finding (in Japan, PCR retesting is not required for discharge if the COVID-19 symptoms have resolved 10 days after the first positive PCR finding).

The results of the viral examination were as follows: EBV viral capsid antigen (VCA)-IgM, 25.9; VCA-IgG, 0.7; and Epstein-Barr virus nuclear antigen (EBNA), 0.3; this suggested a primary EBV infection. The patient had a history of infection with the herpes simplex virus, but no history of cytomegalovirus or toxoplasma infection was found on examination (Table 2). We considered that this was a case of IM caused by EBV infection with COVID-19. The patient had not been vaccinated against COVID-19, but her parents whom she lived with had already been vaccinated twice at least one month prior.

**Table 2:** Results of the subsequent serological tests for infectious pathogens The values given inside brackets mean the normal value in our department. EBV VCA: Epstein-Barr virus viral capsid antigen, EBNA: Epstein-Barr virus nuclear antigen, HSV: herpes simplex virus, CMV: cytomegalovirus, HBs Ag: hepatitis B virus surface antigen, IgM: immunoglobulin M, IgG: immunoglobulin G.

Pathogen-specific antibodies/antigens			
EBV VCA-IgM	25.9	times	(<0.5)
EBV VCA-IgG	0.7	times	(<0.5)
EBNA-IgG	0.3	times	(<0.5)
HSV-IgM	<0.80	times	(<0.80)
HSV-IgG	128	times	(<2.0)
CMV-IgM	<0.85	times	(<0.85)
CMV-IgG	<6.0	times	(<6.0)
Toxoplasma-IgM	<0.50	times	(<0.50)
Toxoplasma-IgG	<1.6	times	(<1.6)
HBs Ag	Negative		(Negative)

## Discussion

IM is thought to be primarily due to overreaction of cell-mediated immunity due to primary saliva-mediated EBV infection. Typical cases among adults include tonsillitis with fever and pseudomembrane formation, cervical lymphadenopathy, and hepatosplenomegaly. By contrast, infants have a weak immune response and often remain asymptomatic or exhibit nonspecific upper respiratory tract inflammation. In addition to EBV, IM may be exhibited not only due to cytomegalovirus but also through other herpesviruses [7]. Although there is currently no reliable treatment, it is generally a disease with a good course and is mostly managed through symptomatic treatment. Antibiotic treatment is sometimes used when the disease is in combination with a bacterial infection, but it is widely known that oral administration of ampicillin causes a rash.

EBV becomes latent after such overt or subclinical infection such as IM is reactivated by signals of proliferation and differentiation of host cells and repeatedly infects the next host cell. Among healthy individuals, this cycle of latency and reactivation is maintained at homeostasis; however, when immunity becomes less effective due to HIV infection or organ transplantation, EBV reactivation or abnormal proliferation of infected cells becomes induced. This has been suggested to be a factor in the development of autoimmune diseases and malignant tumors.

With the COVID-19 pandemic, clinical studies and cases have been conducted in various related fields, with some reports on EBV infection and reactivation. According to Xie et al. and Simonnet et al., EBV reactivation occurred in 17/128 (13.3%) and 28/34 (82.4%) of cases, respectively, in studies on patients with COVID-19 [A1] who were hospitalized in the intensive care unit [1,2]. When not limited to the intensive care unit, EBV reactivation occurred in 68/185 (36.8%) and 37/67 (55.2%) of patients in the studies by Gold et al. and Chen et al., respectively [3,4]. Since the observation period, participants [A2], and the definition of reactivation differ across various studies, the numerical value of the reactivation rate is not constant; nevertheless, EBV reactivation in COVID-19 cases is not rare. According to Xie et al., the EBV-positive group in their cohort had significantly higher respiratory failure, incidence of hypoproteinemia, and mortality rates of 14 and 28 days after admission than the EBV-negative group and required immune-supportive care such as immunoglobulin [1]. EBV reactivation is also reportedly associated with COVID-19 severity.

In the present case, the COVID-19 severity was mild. Serology results showed that the patient likely had an acute EBV infection rather than reactivation. García-Martínez et al. reported a case of SARS-CoV-2 and EBV coinfection in a 19-year-old French woman who received symptomatic treatment, similar to our case [5]. Fukuda et al. also reported an IM case as an atypical symptom of COVID-19 [6]. In their case report, similar to the typical IM caused by EBV, an increase in liver deviation enzyme levels and a marked increase in atypical lymphocyte count were observed. Nevertheless, they have been unable to confirm new infections such as EBV and cytomegalovirus, and a positive finding of PCR test for SARS-CoV-2 was obtained on day seven of hospitalization.

IM is a self-limiting disease that is relieved by follow-up and symptomatic treatment in many cases, but it may sometimes present with splenic rupture due to severe splenomegaly, severe hepatitis, and central nervous system symptoms as complications [8]. Young individuals without a disease history are generally considered to have a lower risk of COVID-19 aggravation; nevertheless, some patients do not exhibit the typical symptoms of COVID-19. In particular, in cases wherein COVID-19 has not converged, it is necessary to still consider the possibility of SARS-CoV-2 infection regardless of the presence or absence of EBV infection, despite observing only symptoms suggestive of IM.

## Conclusions

During the COVID-19 pandemic, we recommend that not only the reactivation of EBV in severe cases of COVID-19 but also the possibility of a SARS-CoV-2 coinfection should be considered in mild and asymptomatic cases among young individuals, despite being preceded by symptoms suggestive of IM.
